The article "Cardiovascular Disease and Exercise: From Molecular Mechanisms to Clinical Applications" was retracted in 2023. Reason: plagiarism.

# Cardiovascular Disease and Exercise: From Molecular Mechanisms to Clinical Applications

**DOI:** 10.3390/jcm11247511

**Published:** 2022-12-19

**Authors:** Bo Wang, Lin Gan, Yuzhi Deng, Shuoji Zhu, Ge Li, Moussa Ide Nasser, Nanbo Liu, Ping Zhu

**Affiliations:** 1 Guangdong Cardiovascular Institute, Guangdong Provincial People’s Hospital, Guangdong Academy of Medical Sciences, Guangzhou 510100, China; xnwangbo430@hotmail.com (B.W.); ganganm3@126.com (L.G.); 18975612968@163.com (Y.D.); zhushuoji@gmail.com (S.Z.); lige5@mail.sysu.edu.cn (G.L.); 2 Guangdong Provincial Key Laboratory of Pathogenesis, Targeted Prevention and Treatment of Heart Disease, Guangzhou 510640, China

**Keywords:** exercise factor, cardiac protection, mitochondria, insulin sensitivity, exercise prescription, cardiac rehabilitation

## Abstract

Inactivity is a significant risk factor for cardiovascular disease. Exercise may greatly enhance the metabolism and function of the cardiovascular system, lower several risk factors, and prevent the development and treatment of cardiovascular disease while delivering easy, physical, and emotional enjoyment. Exercise regulates the cardiovascular system by reducing oxidative stress and chronic inflammation, regulating cardiovascular insulin sensitivity and the body’s metabolism, promoting stem cell mobilization, strengthening autophagy and myocardial mitochondrial function, and enhancing cardiovascular damage resistance, among other effects. Appropriate exercise intervention has become an essential adjuvant therapy in clinical practice for treating and rehabilitating various cardiovascular diseases. However, the prescription of exercise for preventing and treating cardiovascular diseases, particularly the precise selection of individual exercise techniques and their volume, remains controversial. Using multiomics to explain further the molecular process underlying the positive effects of exercise on cardiovascular health will not only improve our understanding of the effects of exercise on health but also establish a scientific basis and supply new ideas for preventing and treating cardiovascular diseases by activating the endogenous protective mechanisms of the body and suggesting more specific exercise prescriptions for cardiovascular rehabilitation.

## 1. Introduction

The beneficial effects of exercise on cardiovascular health are generally recognized, but the mechanisms underlying their benefits remain obscure. Physical activity boosts cardiovascular health by a systemic action, including the metabolism of neurons and endocrine, immunological, and other systems [1,2]. The essence of this effect is the activation of endogenous protective mechanisms due to a lack of oxygen, oxidative stress, and mechanical force stimulation (such as flow acceleration), such as the activation of cell survival signals, which upregulate the body’s metabolism, enhance the antioxidant capacity and promote stem cell mobilization.

The article "Cardiovascular Disease and Exercise: From Molecular Mechanisms to Clinical Applications" was retracted in 2023. Reason: plagiarism.

Mitochondria are vital organelles that mediate the body’s response to movement. The promotion of mitochondrial synthesis and enhancement of mitochondrial function through signalling molecules such as peroxisome proliferator-activated receptor-coactivator-1 (PCC-1) is essential for the health benefits of exercise [3,4]. According to Wang et al. [5], cardiomyocyte apoptosis and vascular endothelial dysfunction might result in detrimental cardiovascular system remodeling, leading to the onset and progression of IHD. Exercise intervention primarily activated the PI3K/Akt pathway, raised the amount of anti-apoptotic factors, decreased pro-apoptotic factors, and greatly lowered cardiomyocyte apoptosis and unfavorable remodeling. By activating the PI3K/Akt/eNOS pathway, the level of NO can be increased, endothelial cell proliferation and migration can be stimulated, damaged endothelial cells can be repaired, the vascular endothelial function can be enhanced, the progression of IHD can be stabilized, and the disease state can even be reversed. Similarly, moderate aerobic exercise (16 m/min, 60 min/d, 5 days/wk) can activate the neuregulin-1 (NRG1)/epidermal growth factor receptor, ErbB, and fibroblast growth factor 21 (FGF21)/PI3K/AKT to inhibit myocardial apoptosis, reduce the MI area, reduce myocardial fibrosis, and promote cardiac repair and angiogenesis, and improve heart disease’s rational remodeling and cardiac function [6]. Whereas, long-term and intensive aerobic activity may cause physiological hypertrophy of the heart and thereby enhance cardiac function. In contrast to pathological hypertrophy, physiological hypertrophy is not accompanied by pathological changes such as cardiac fibrosis. This type of exercise strongly triggers the IGF1-PI3K-Akt signalling pathway in the myocardium [7] (Figure 1).

In addition, exercise may lower cardiovascular disease risk factors, modify the cardiovascular structure and function, and enhance insulin sensitivity and loss resistance, among other effects. Exercise-related molecule production by numerous tissues and organs contributes to metabolism and cardiovascular protection, highlighting the relevance of crosstalk between tissues and organs in the exercise-induced improvement of cardiovascular health. This paper briefly introduces the current paradigm of the clinical prevention and treatment of cardiovascular disease through exercise.

## 2. Exercise Reduces the Risk Factors for Cardiovascular Disease and Its Main Mechanism

### 2.1. Exercise Improves the Body’s Metabolism

Metabolic syndrome, which is characterized by obesity, hyperlipidemia, impaired glucose tolerance, and insulin resistance, is a major risk factor for cardiovascular diseases, including hypertension, atherosclerosis, and coronary heart disease. Various forms of exercise may improve glucose, lipid, and insulin sensitivity [8]. The molecular benefits include significantly lowered triglycerides, increased high-density lipoprotein levels, accelerated browning and thermogenesis in adipose tissue, enhanced fatty acid metabolism, increased muscle mass, and decreased body fat. A recent study has shown that the metabolic imbalance of amino acids is a major cause of cardiovascular and metabolic illness. Exercise may alleviate the metabolic problem of basal and branched-amino acids (BCAA) in pathological situations such as diabetes by increasing the cellular usage of amino acids and consequently enhancing cardiovascular, cardiometabolic, and metabolic health [9,10,11,12,13].

The article "Cardiovascular Disease and Exercise: From Molecular Mechanisms to Clinical Applications" was retracted in 2023. Reason: plagiarism.

### 2.2. Exercise Improves REDOX Balance and Chronic Inflammatory State

The underlying pathophysiological cause of numerous cardiovascular diseases is oxidative stress. Long-term exercise may improve the redox state of the body by boosting the antioxidant capacity, which is one of the most important processes through which exercise enhances cardiovascular health. During physical exercise, the contraction of skeletal muscle increases the generation of reactive oxygen species (ROS), which are primarily generated by the mitochondrial electron transfer pathway [14,15,16]. ROS might cause cellular oxidative stress and are a type of active hazardous material that causes biological macromolecular damage. The production of adequate ROS is physiologically necessary. ROS generated during exercise may stimulate mitochondrial synthesis, activate insulin signalling, stimulate protein synthesis and muscle development, control gene expression, and boost the body’s antioxidant capacity. Long-term exercise may improve mitochondrial function, the body’s antioxidant capacity, and the maintenance of its oxidative level [17]. Suppressing ROS generation during exercise reduces the health benefits of exercise [18]. Exercise may also improve mitochondrial dynamics by suppressing excessive mitochondrial division in cardiovascular disorders (ischaemic heart disease, heart failure) [19]. Acute exercise may have a similar “ischaemic preconditioning” effect on the heart by increasing the cardiac mitochondrial formation of ROS. Long-term physical activity may improve the mitochondrial antioxidant capacity and heart REDOX status [20,21]. Both aerobic exercise and resistance exercise substantially influence the homeostasis and function of mitochondria and are essential to the benefits of exercise on cardiovascular health.

The article "Cardiovascular Disease and Exercise: From Molecular Mechanisms to Clinical Applications" was retracted in 2023. Reason: plagiarism.

Numerous chronic diseases, particularly metabolic cardiovascular disorders, throw the body into a state of low-grade chronic inflammation, which results in chronic non-communicable diseases (NCDs) and represents a significant cause of chronic diseases and accelerated ageing. Long-term aerobic exercise was reported to decrease chronic inflammation and is an effective technique for interrupting this vicious cycle. Similarly, previous studies have shown that aerobic exercise may reduce the inflammatory marker high-sensitivity C-reactive protein (hS-CRP) by 40% in coronary heart disease patients [22]. Additionally, exercise may boost the synthesis of interleukin-6 (IL-6) in human skeletal muscle and reduce the production of tumour necrosis factor-α (TNF-α), interleukin-1 (IL-1), and other proinflammatory molecules, and exercise thus serves as an anti-inflammatory input [23]. Furthermore, exercise may enhance fat metabolism, reduce visceral fat, and activate the hypothalamic–pituitary–adrenal axis and sympathetic nervous system to generate cortisol and other anti-inflammatory cytokines [24]. Long-term exercise has a systemic influence on the redox balance and inflammatory state of the body and may enhance cardiovascular health directly or indirectly.

### 2.3. Exercise Slows Ageing

The ageing process is associated with structural and functional body changes and is a risk factor for chronic diseases such as cardiovascular disease. Long-term and consistent aerobic activity exerts an antiageing effect because it may encourage the migration of stem cells, resulting in a “youthful” body [25]. Exercise, for example, decreases the activation of glial cells due to ageing and increases the glial cell volume by increasing the levels of insulin-like growth factor 1 (IGF1) and the vascular endothelial growth factor (VEGF). These growth factors boost the central nervous system’s insulin sensitivity and promote neurogenesis and angiogenesis. These activities may enhance cerebral blood flow, reduce amyloid deposition, and delay age-related neurodegenerative changes [26]. Exercise may also enhance the ageing-related endocrine function of the hypothalamic–pituitary axis and the muscular and bone condition of elderly individuals [27]. The effects of exercise on heart ageing include the following:

✓ Senile heart β adrenoceptor desensitization makes the heart less sensitive to adrenergic stimulation. Exercise can enhance the sensitivity of the myocardium to adrenergic stimulation and thus increases the cardiac functional reserve [28].
✓ The heart loses its Ca^2+^ processing capacity as it ages. The same stimulation reduces the intracellular Ca^2+^ increase and the cell contractility. Exercise can enhance intracellular Ca^2+^ processing capacity and cell contractility [29].

The article "Cardiovascular Disease and Exercise: From Molecular Mechanisms to Clinical Applications" was retracted in 2023. Reason: plagiarism.

Mitochondrial dysfunction is an important mechanism for modulating cardiac function, in which exercise improves mitochondrial dynamics and function to adjust the cardiac metabolism, reduce oxidative stress, and increase the cardiac reserve capacity [30]. Moreover, vascular ageing is typically characterized by thickening and stiffening of large blood vessel walls, endothelial dysfunction, thrombosis-promoting changes in the vascular endothelium, proinflammatory and vasoconstrictive phenotype transformation, smooth muscle to secretory type changes, and reduced angiogenesis ability [31]. Long-term aerobic exercise can ease and even partly reverse the vascular ageing alterations listed above [32]. The fundamental mechanism through which exercise prevents ageing might be increasing the body’s antioxidant capacity and redox state because oxidative stress is a major cause of ageing.

### 2.4. Exercise Prevention and Treatment of Hypertension

Numerous scientific and clinical studies have shown that physical activity helps prevent and cure hypertension. Scientists have reported that all exercises (such as endurance, dynamic resistance, and isometric muscular strength training) reduce systolic blood pressure. Regular aerobic exercise may lower the resting blood pressure of hypertensive individuals by 57 mm Hg [33]. Similarly, high-intensity interval training and continuous aerobic training have similar effects on lowering blood pressure. Still, high-intensity interval training has tremendous potential for enhancing cardiopulmonary endurance, vascular endothelial function, and insulin sensitivity [34,35]. It is currently believed that the mechanism through which exercise prevents and improves hypertension consists primarily of the following:

✓ Reducing the resting systolic.
✓ Improving the oxidative stress levels and regulating the renin–angiotensin system to affect vascular remodelling and blood vessels.
✓ Increasing insulin sensitivity and nitric oxide (NO) bioavailability and promoting vasodilation and tissue perfusion.

### 2.5. Muscle-Building Effects of Exercise and Cardiovascular Health

Skeletal muscle represents approximately 40% of the human body’s mass, which makes it the most conspicuous organ. In addition to carrying out the body’s motor function, skeletal muscle is one of the major organs involved in glucose metabolism and, by extension, glucose homeostasis. A decrease in skeletal muscle mass may impair glucose metabolism and tolerance. In addition to enhancing insulin sensitivity, the muscle-building effect of exercise promotes glucose metabolism and tolerance by enhancing blood glucose “pathways” (into the skeletal muscle) that serve to buffer increases in blood glucose. Moreover, muscle is an essential endocrine organ of the body that can regulate cardiovascular metabolism and function via the production of various exercise factors. Recently, it has shown an association between the amount of human muscle tissue and the incidence and mortality of cardiovascular disease [36,37]. Muscular atrophy (e.g., sarcopenia) is characterized by a decrease in muscle-derived carnitine, which is essential for fatty acid transport in the heart and skeletal muscle and thus leads to abnormal fatty acid metabolism. Sarcopenia is common in patients with heart failure due to the retention of the ejection fraction, which may result in cardiovascular dysfunction due to abnormal glucose and lipid metabolism and decreased production of exercise hormones [38,39].

The article "Cardiovascular Disease and Exercise: From Molecular Mechanisms to Clinical Applications" was retracted in 2023. Reason: plagiarism.

### 2.6. Other

In recent years, many studies have investigated the mechanism through which the biological function of gut bacteria can influence cardiovascular health via their metabolites. Indeed, the time it takes for physical exercise to affect intestinal flora is linked to higher body fat, higher triglycerides, and better circulation of high-density lipoprotein cholesterol (HDL-c) and blood pressure. Intriguingly, the intestinal microbiota of top athletes and inactive individuals exhibit metagenomic and metabolomic differences, which shows that regular exercise might enhance metabolic health by improving the intestinal microbiota [40,41,42]. For instance, Liu et al. reported that exercise may boost short-chain fatty acids and decrease branched-chain amino acid (BCAA) levels by enhancing the gut flora and thus improve glucose metabolism and insulin sensitivity [43]. Also, mental and psychological variables contribute to the onset and progression of ischaemic heart disease. Exercise may alleviate psychological stress, lower the moderate=to-severe anxiety prevalence in coronary heart disease patients by 56% to 69%, and facilitate cardiac rehabilitation [44]. In addition, physical activity may increase stem cell mobilization and tissue healing [45]. These interactions are principal contributors to cardiovascular health (Figure 2).

## 3. Exercise Improves the Cardiovascular Structure and Function

### 3.1. Remodeling of the Cardiovascular Structure and Function

Even moderate exercise reduces pathological ventricular hypertrophy, such as that caused by heart failure, and improves cardiac shape and function under pathological conditions. Exercise-induced vascular remodelling is characterized by increases in the arterial vessel diameter and arterial vessel wall thickness (including coronary arteries) [46]. Likewise, exercise increases collagen and elastin content in atherosclerotic plaques while decreasing atherosclerosis-related adverse outcomes [47]. This effect may be one of the mechanisms through which physical activity protects vital organ function and retards ageing [48].

The article "Cardiovascular Disease and Exercise: From Molecular Mechanisms to Clinical Applications" was retracted in 2023. Reason: plagiarism.

Exercise impacts blood vessels and increases the development of new blood vessels. Exercise, may increase the capillary formation and promote angiogenesis, while it may widen the arterial lumen through a process known as arteriogenesis (Figure 3). This process may occur in existing blood vessels (including coronary arteries) and thus demonstrates substantial vascular system adaptability. A key regulator of angiogenesis is the vascular endothelial growth factor (VEGF), whose expression in skeletal and cardiac muscle may be increased by exercise [49,50].

Conversely, in atherosclerosis, exercise may enhance the amount of circulating endostatin and angiogenesis in plaque tissue, thus preventing the progression of atherosclerotic plaque, which may have important implications for the prevention and treatment of coronary heart disease [51]. However, certain circumstances are required for angiogenesis and arteriogenesis to maintain tissue perfusion. The disturbance of these systems is one of the pathogenic mechanisms underlying several diseases, such as coronary heart disease. Angiogenesis and arteriogenesis may boost coronary collateral circulation, reduce myocardial damage during myocardial infarction, and improve blood perfusion and tissue healing [52]. Exercise may stimulate the ischaemic myocardium, and angiogenesis and arteriogenesis can increase coronary collateral circulation and improve blood vessel and tissue healing perfusion. Endothelial dysfunction is one of the pathogenic mechanisms contributing to the development and progression of certain cardiovascular diseases. Physical activity may improve vascular endothelial function through mechanisms independent of cholesterol, blood pressure, glucose tolerance, and body weight [53].

The effect of exercise on cardiovascular health is partially attributable to its direct mechanical stimulation of the cardiovascular system. One of the primary variables of cardiovascular function is mechanical force. For example, exercise-induced acceleration of the tissue blood flow increases shear forces, stimulating nitric oxide generation by vascular endothelial cells, widening capillaries, and improving blood perfusion to tissues and organs [54]. Similarly, shear stress-induced movement increases blood flow and can directly induce vascular endothelial cells to secrete a movement factor. The latter, which is absorbed by heart muscle cells from outside the blood circulation and plays a role in cardiac protection, promotes interactions between the heart and blood vessels to affect cardiovascular regulation and protection [55]. In a recent population-controlled study, stretching was found to be more effective for lowering blood pressure than brisk walking. The process may be related to the enhancement of vascular stiffness by mechanical stretching stimulation [56].

The article "Cardiovascular Disease and Exercise: From Molecular Mechanisms to Clinical Applications" was retracted in 2023. Reason: plagiarism.

The mechanism through which mechanical force stimulates and garners a response in the cardiovascular system remains unknown. Piezo receptors on the cell membranes of vascular endothelial cells, smooth muscle cells, and other tissues may sense mechanical force stimulation and initiate cellular calcium influx, resulting in changes in cellular functional activities. These receptors regulate cardiovascular function in response to exercise and are linked to the initiation and progression of cardiovascular diseases such as atherosclerosis, heart failure, and hypertension [57,58].

### 3.2. Improvements in Myocardial Mitochondrial Function and Metabolism

Numerous studies have shown that increased mitochondrial activity is directly connected to the cardioprotective benefits of exercise. Mitochondria govern metabolic, redox, and cell fate processes. The myocardium is the most mitochondrially dense tissue in the body, accounts for approximately 40% of the volume of cardiomyocytes, and serves as the heart’s main energy source. During exercise, the energy demands of the heart increase substantially, leading to an increase in ATP generation. In addition, the heart has access to almost all metabolic substrates. Under normal conditions, the major metabolic substrate of the heart is lipoic acid (40–70%). During exercise, the myocardium increases its use of fatty acids and lactic acid while decreasing its glucose usage. Prolonged exercise increases myocardial glucose use, particularly the glycolysis level, which is related to the establishment and progression of cardiac physiological hypertrophy [59,60]. Under normal conditions, the major metabolic substrate of the heart is lipoic acid (40–70%). During exercise, the myocardium increases its use of fatty acids and lactic acid while decreasing its glucose usage. Prolonged exercise increases myocardial glucose use, especially the glycolysis level, which is related to the establishment and progression of cardiac physiological hypertrophy [61,62]. Long-term exercise may increase mitochondrial dynamics and function and thus increases the pace and efficiency of cardiac metabolism and the adaptability of the metabolic switch and strengthen myocardial damage resistance [63]. Exercise increases the transcription factors PGC-1, PPAR, NRF2, and others that govern cell function and mitochondrial homeostasis [64].

The article "Cardiovascular Disease and Exercise: From Molecular Mechanisms to Clinical Applications" was retracted in 2023. Reason: plagiarism.

### 3.3. Other

In addition to the abovementioned mechanisms, exercise influences cardiovascular function. For example, prolonged hyperexcitation of sympathetic neurons has a negative impact on the structure and function of the cardiovascular system, which is one of the causes of several cardiovascular diseases [65]. Long-term aerobic exercise may enhance cardiovascular autonomic nervous system function and homeostasis, increase parasympathetic nerve activity, decrease sympathetic nervous activity, increase heart rate variability (HRV), thereby exerting a cardioprotective effect. Cardiorespiratory fitness (CRF) reduction due to ageing or long-term inactivity is also connected to the onset and development of cardiovascular diseases. According to a meta-analysis, all-cause mortality and cardiovascular mortality are lowered by 13 and 15%, respectively, for each additional metabolic equivalent (MET) of cardiopulmonary fitness [66,67]. Aerobic and resistance exercise may improve both cardiorespiratory fitness and cardiovascular health.

## 4. Exercise-Related Factors and Cardiovascular Protection

Exercise exerts a systematic and comprehensive effect on health. Exercise not only produces a direct effect locally in organs or tissues, but also induces the expression of exercise factors in these organs and tissues. Exercise factors are bioactive compounds, such as peptides or nucleic acids, that are produced by skeletal muscles and other organs to carry out the biological effects of exercise [68]. The understanding of exercise factors has been refined over the years. These factors are a class of bioactive compounds produced or increased by training in several tissues and organs and may be proteins and nucleic acids or very small molecules, such as metabolites, that act through endocrine or paracrine processes on the same or other tissues and organs. Exercise factors influence the development of tissues and organs, physiological function, and overall health. Considering them as a whole, we believe that exercise elements should have the following three key characteristics:

✓ Bioactive substances produced during exercise or promoted by exercise.
✓ Release from cells to adjacent cells or into the blood circulation to act on other organs or tissue cells.
✓ Affect the growth or functional activity of recipient cells and thus usually mediate the health effects of exercise.

The article "Cardiovascular Disease and Exercise: From Molecular Mechanisms to Clinical Applications" was retracted in 2023. Reason: plagiarism.

Exercise factors (such as IL-6 and irisin, etc.) discovered in the early stage are mainly derived from skeletal muscle proteins called myokines. In recent years, new exercise factors have been discovered and reported, and their sources include fat, liver, vascular endothelial cells, and other tissue cells.

### 4.1. Muscle Factors

Muscle factors are a class of bioactive cytokines that are secreted by skeletal muscle during and after exercise. Among the primary processes through which exercise enhances cardiovascular health are the activity of muscle factors on the tissues and organs of the whole body through endocrine or paracrine pathways. Myostatin was the first muscle factor discovered to activate SMAD (an acronym from the fusion of Caenorhabditis elegans Sma genes and the Drosophila Mad, Mothers against decapentaplegic) signalling and inhibit mammalian target of rapamycin (mTOR) signalling. Exercise can reduce the expression of myostatin, which is associated with the reduction of fat content, the promotion of white fat browning and good muscle weakness. While an increased myostatin expression in cardiomyocytes in heart failure has a cardioprotective effect, it is also one of the causes of skeletal muscle atrophy in heart failure [69,70]. 

IL-6 is the most often reported muscle factor. Exercise promotes the synthesis of IL-6 in skeletal muscle, which is essential for exercise-mediated metabolic remodelling and anti-inflammatory effects. IL-6 may enhance glucose and fatty acid metabolism by stimulating the AMPK signalling system in skeletal muscle and fat. This cytokine may also increase the synthesis of anti-inflammatory molecules such as IL-10 and sTNF-R and reduce the release of proinflammatory factors such as TNF-α. Additionally, IL-6 increases muscle growth and angiogenesis. Exercise has also been linked to the interleukin family members IL-15, IL-7, IL-8, IL-4, and IL-13, in addition to IL-15, IL-7, IL-8, and IL-13 [71,72,73].

Exercise increases the expression and cleavage of fibronectin type III domain-containing protein 5 (FNDC5) by activating the PGC-1α signalling pathway in skeletal muscle. FNDC5 is secreted by skeletal muscle cells after the cleavage of irisin. Irisin mainly enhances mitochondrial activity by activating signalling mechanisms such as the MAPK and uncoupling protein-1 (UCP-1) pathways in target cells and generates various biological responses, such as promoting myocardial regeneration and angiogenesis. Improved endothelium-dependent and non-endothelium-dependent vasodilation and reduced myocardial fibrosis exert protective effects on heart failure, myocardial ischaemia/reperfusion injury, and other vascular diseases [74]. In addition to these factors, some other myofactors, such as meteorin-like protein (METRNL) and follistatin-like 1 (FSTL1), reportedly improve endothelial function and promote vascular regeneration by activating eNOS [75]. Apelin can improve insulin sensitivity, support vasodilation, enhance myocardial contractility, and promote angiogenesis to protect cardiovascular function [76,77]. Myonectin promotes fatty acid metabolism. Musclin promotes mitochondrial biosynthesis and inhibits glucose uptake in skeletal muscle. Previously, these myofactors were all thought to be encoded by nuclear genes. Recent studies have found that MOTS-c, which is encoded by mitochondrial genes, is also a motor factor that can promote the body’s motor function [78]. In addition to the abovementioned proteins, some small-molecule metabolites (such as aminobutyric acid) and nucleic acids secreted by skeletal muscle may also be directly or indirectly involved in cardiovascular-protective effects (Figure 4) [79].

The article "Cardiovascular Disease and Exercise: From Molecular Mechanisms to Clinical Applications" was retracted in 2023. Reason: plagiarism.

### 4.2. Adipose Factor

In addition to releasing cytokines, adipose tissue is capable of releasing adipokines. Exercise may affect the production and secretion of a variety of adipokines, particularly by boosting the secretion of adiponectin and reducing that of leptin. Adiponectin, which is one of the most extensively studied adipokines to date, can stimulate the utilization of fatty acids and glucose in skeletal muscle, inhibit hepatic gluconeogenesis and the production of the proinflammatory macrophage factor TNF-α, and stimulate the production of the anti-inflammatory factor IL-10 [80]. 

Hypoadiponectinemia is associated with metabolic diseases such as type 2 diabetes, coronary heart disease, and high blood pressure. Adiponectin prevents cardiac hypertrophy, decreases apoptosis by activating AMPK, and has anti-inflammatory effects by augmenting COX-2 expression [81,82]. Leptin is a well-researched adipokine that controls the body’s fat content and metabolism. High leptin levels are strongly associated with atherosclerosis, hypertension, and other cardiovascular disorders. Likewise, leptin causes inflammation, promotes the transformation of smooth muscle cell proliferation and the smooth muscle phenotype, and activates the sympathetic nervous system, among other effects [83]. 

### 4.3. Noncoding RNA

Exercise can affect the expression of a variety of noncoding RNAs (ncRNAs). These ncRNAs can exert a biological effect in cells and can be secreted to act on distant cells [84,85]. In recent years, a growing number of studies have shown that exercise affects ncRNAs. It has been reported that changes in the expression of the microRNAs (miRNAs) mir-1, mir-133a, and miR761 in skeletal muscle after exercise can promote the expression of the skeletal muscle metabolism-related proteins MAPK and PGC-1α and thereby improves the body’s metabolism and the anti-injury ability of the heart [86]. Exercise promotes mir-16 production by neutrophils; mir-17 and mir-18a are involved in various inflammatory reactions [87]. Exercise is involved in the occurrence and progression of cardiac physiological hypertrophy after exercise by regulating the expression of miR-143, miR-124, and miR1145 [88,89]. However, exercise can reduce myocardial injury after cardiac ischaemia/reperfusion injury by inhibiting the abnormal expression of miR-214, miR-1, and miR-29a [90,91]. MALAT1 is a long noncoding RNA (lncRNA) that is elevated in diabetes mellitus, can contribute to insulin resistance, and participates in the development of diabetes, and exercise can reduce MALAT1 and improve the metabolic abnormalities of diabetes [92]. These findings indicate that ncRNAs are widely involved in exercise-induced cardiovascular physiological and pathological processes.

The article "Cardiovascular Disease and Exercise: From Molecular Mechanisms to Clinical Applications" was retracted in 2023. Reason: plagiarism.

## 5. Exercise Improves Insulin Sensitivity and Loss Resistance in the Cardiovascular System

The underlying pathophysiology of hypertension, coronary heart disease, diabetes, and other cardiovascular disorders is insulin resistance [93,94]. A lack of physical exercise is directly related to impaired glucose tolerance, a crucial clinical sign of diabetes mellitus, and numerous cardiovascular and metabolic diseases. Exercise may increase insulin sensitivity in both insulin-sensitive and insulin-resistant individuals. Studies indicate that both short- and long-term exercise may significantly improve insulin sensitivity. In fact, exercise can reverse the molecular defects in several areas of the insulin signalling system [95,96]. This effect extends for 16 to 48 h after intense activity. Long-term, regular physical exercise may improve glucose absorption and metabolism in both normal and diabetic individuals [97,98].

Previous research on insulin sensitivity has mainly focused on the whole body and the principal organs targeted by insulin, such as skeletal muscle, liver, and fat. Very few studies have focused on insulin sensitivity in the cardiovascular system. Myocardial and vascular insulin resistance may occur independently of systemic insulin resistance and are tightly linked to the development of cardiovascular dysfunction and other cardiovascular diseases [99,100]. In the early phase of myocardial ischaemia, for example, a TNF-α-driven inflammatory response may result in myocardial insulin resistance and thus contributes to the start and progression of ischaemic heart failure [101]. Prehypertension is associated with vascular insulin resistance, which leads to vascular dysfunction and hypertension [102]. Along with improving chronic cardiovascular inflammation and insulin sensitivity, aerobic exercise may reduce cardiovascular risk factors such as hyperglycemia, hyperlipidaemia, and obesity and improve cardiovascular health and protection [103,104]. Similarly, exercise increases circulatory function and cardiovascular resistance to injury. Indeed, a single exercise session may prevent future cardiac ischaemia–reperfusion damage, and those habitual exercisers can preserve this cardioprotective benefit for months after stopping exercise [105]. 

The article "Cardiovascular Disease and Exercise: From Molecular Mechanisms to Clinical Applications" was retracted in 2023. Reason: plagiarism.

## 6. Application of Disease Treatment and Rehabilitation in Heart Vessel Disease

An appropriate exercise intervention substantially impacts cardiovascular disease, and guidelines provide specific recommendations for various cardiovascular disorders. Numerous challenges remain in preventing and treating blood vessel damage and rehabilitating heart disease patients. Heart failure (HF) is the terminal phase of some heart diseases. Due to cardiac insufficiency and exercise intolerance, the physical activity of HF patients is severely restricted, which is presently considered outmoded and inappropriate [106,107,108]. Even those with severe cardiac problems, such as HF, may benefit from modest exercise. Patients with stable HF must participate in physical exercise as an adjunct to their HF therapy and as a necessary treatment. Before recommending exercise to individuals with HF, the individuals must undergo a thorough medical assessment that should concentrate on three major factors:

✓ Patients with exercise contraindications, such as hypotension or hypertension during quiet or exercise, unstable or worsening disease, significant myocardial ischaemia or concomitant serious lung disease, etc., were excluded (not recommended to practice long-term exercise).
✓ The basic functional assessment includes comprehensive detection of cardiac function, complications, maximum exercise capacity, and risk assessment. Optimized treatment plans and standard treatment should be given to patients with heart failure [109].
✓ The cardiopulmonary exercise test is essential for determining a patient’s maximal exercise capacity to determine an appropriate training intensity and modality [110].

The heart failure clinical trial findings demonstrate that moderate-intensity exercise may greatly increase the maximal exercise capacity of patients with heart failure and that the more exercise performed, the larger the benefits [111,112]. In contrast, exercise has no adverse effects on defibrillator-implanted patients with heart failure. Therefore, aerobic exercise is recommended for the majority of individuals with heart failure [113]. 

The article "Cardiovascular Disease and Exercise: From Molecular Mechanisms to Clinical Applications" was retracted in 2023. Reason: plagiarism.

The combination of endurance and resistance training produces more substantial benefits. Resistance training is more suitable for HF patients with a low-risk profile and improves the muscle status and body stability of older people. Resistance training may also be used as a supplement to aerobic exercise. In addition, the exercise regimen of a person with HF must account for the various types of HF. In recent years, exercise prescriptions for coronary heart disease, hypertension, and diabetes, among other diseases, have climbed alongside those for HF. Due to the diversity between humans and the complexity of exercise training, several barriers remain to generating effective exercise prescriptions for patients with cardiovascular disease [114,115,116].

## 7. Discussion and Prospects

Although the influence of exercise on cardiovascular health has been well established, methods for enhancing these benefits remain obscure. Its therapeutic use is mostly limited to cardiac rehabilitation and lacks a specific direction. Indeed, the local effects of exercise on a single tissue or organ, and research on the integrated process underlying the health benefits of exercise, are lacking. With the development and maturity of various integrated research approaches and multiomics technologies, studies based on the effect-multiomics-molecular-function paradigm will provide fresh insights into the whole mechanism of the effects. The significance of multidimensional omics research methodologies (such as multiomics, multiorgan, and time–space coupled applications) will increase.

It is essential to evaluate whether the type and intensity of exercise undertaken by different groups or patients provide the greatest health advantages. Several studies have explored the effects of different forms of exercise on physical health and determined that the health advantages of training depend on the exercise method, and team activities typically give greater health benefits [117,118,119]. Low- and moderate-intensity exercise greatly reduces the risk of cardiovascular disease and increases metabolism, but high-intensity exercise significantly improves cardiopulmonary fitness. Similarly, the functional improvement and health effects associated with high-intensity exercise are more pronounced under certain exercise conditions, which suggests that the biological effects of different exercise intensities may differ when all other conditions are equal, although the exact mechanism is unknown [120]. The selection of the exercise mode and intensity based on age and physical condition is an essential component of public fitness. Regardless of any type, intensity, or age, exercise could increase the heart rate and blood flow benefits health. However, fitness and exercise should conform to the basic “Listen to your body” guideline. Under different physiological or pathological conditions (such as hypertension, diabetes, and heart failure) and in elderly individuals, it is essential to appropriately identify the exercise intensity, and this is a particular focus of clinical cardiovascular rehabilitation specialists and is also one of the top research objectives and problems in sports medicine. In addition, the influence of the biorhythm on human physiological and pathological processes has received significant attention in recent years; the periodicity of fitness exercise, i.e., the time of day when they may gain the maximum health advantages. Indeed, afternoon exercise has better glycaemic and health effects on people with diabetes than morning exercise [121].

The article "Cardiovascular Disease and Exercise: From Molecular Mechanisms to Clinical Applications" was retracted in 2023. Reason: plagiarism.

The duration of the health advantages of exercise is uncertain. Indeed, long-term exercise may have long-term health implications through epigenetic modification. A recent epidemiological study found that adolescents aged 7 to 17 years who exercised for more than 180 min per week for more than 9 months had at least a 50% decreased risk of developing hypertension and type 2 diabetes in old age [122]. In addition, parental involvement enhances their children’s health [123,124,125]. These findings suggest that exercise may have long-term health advantages, but the exact mechanism is unknown. In addition, whether physical exercise at different stages of human development (such as infancy or old age) has distinct health repercussions of distinct magnitudes is a new area of academic interest. In recent years, elucidating the molecular mechanism underlying the health advantages of exercise, mainly via the use of diverse omics approaches, has been a hot topic in exercise health. The cardiovascular health advantages of exercise have a systemic impact. Recent discoveries regarding exercise factors provide a new understanding of the mechanism of exercise-induced health effects, particularly the interaction between tissues and organs. These findings are expected to provide new ideas and strategies for developing new drugs or methods to simulate the health effects of exercise. Clarifying the connection between tissues and organs and the molecular mechanism underlying the health effects of exercise is crucial for generating precise individual exercise prescriptions. This study topic is becoming more prominent and will soon be at the forefront and epicenter of sports health research.

The article "Cardiovascular Disease and Exercise: From Molecular Mechanisms to Clinical Applications" was retracted in 2023. Reason: plagiarism.

After a thorough evaluation, exercise prescriptions should specify the type, frequency, duration, and intensity of exercise. Aerobic, resistance and total-body exercises may be generally characterized; nevertheless, the intensity and frequency of exercise should correspond to the principles of individualization and progression. In individuals with HF whose status is stable after exercise, exercise intervention should be commenced as soon as feasible. During the activity (particularly at the beginning), a physician or other expert should give advice and assessment, including an examination of the heart rate, which is the most popular method for evaluating exercise intensity. During exercise, arrhythmia and abnormal blood pressure should also be recorded. Following the course of the disease and the patient’s state, the exercise regimen for HF patients should be adjusted at least every three to six months. Additionally, efforts should be made to mobilize patients’ enthusiasm to participate in sports training. Regardless, patients with a good attitude and cooperative spirit may have better health results.

Exercise offers great therapeutic potential for preventing and treating cardiovascular disease, but several issues must be clarified. Each person has a unique “endogenous medication arsenal”. In-depth basic research on uncovering and efficiently using the body’s endogenous health resources is urgently needed, particularly research on generating scientific and highly compliant cardiac rehabilitation exercise prescriptions for individuals with various conditions and characteristics. In addition, with the advancement of science related to smart devices and technology, researching the use of modern science and technology, such as various types of smart apparel and big data, for monitoring and optimizing individual sports effects and preventing all types of adverse cardiovascular events caused by excessive movement, among other goals, is of the utmost importance.

The human body has evolved into a complex and potent endogenous defense system throughout evolution, and exercise is one of the most effective triggers for activating this mechanism and maintaining health. Compared to pharmacological cardiovascular disease prevention and treatment, exercise primarily plays a systematic role in cardiovascular protection by activating the body’s endogenous protection mechanism, making exercise a cost-effective, safe, enjoyable, and effective means of promoting cardiovascular health. In fact, the theory and practice of traditional Chinese medicine have emphasized that “exercise is the key to life” for centuries. Clarifying the mechanism through which exercise benefits cardiovascular health, the formulation of individualized, precise exercise prescriptions, and mobilization of the body’s endogenous protection mechanism through moderate exercise are essential strategies and directions for promoting cardiovascular health, preventing cardiovascular diseases, and treating cardiovascular diseases.

The article "Cardiovascular Disease and Exercise: From Molecular Mechanisms to Clinical Applications" was retracted in 2023. Reason: plagiarism.

## Figures and Tables

**Figure 1:** Exercise-induced health effects and central role of mitochondria: Hypoxia, oxidative stress, mechanical force, and other variables play a role in activating endogenous defensive systems when exercise is performed. These endogenous defensive mechanisms include the survival signalling pathways of PI3K-Akt-eNOS-NO and the metabolic signalling pathways of PGC-1-AMPK-mTOR. Mitochondria are an extremely important factor in the positive health impacts of exercise.

**Figure 2:** Exercise-induced cardiovascular benefits and underlying mechanisms: Exercise benefits cardiovascular health through its effects on the body. The primary mechanisms include enhancement of insulin sensitivity and metabolism in the cardiovascular system, reductions in oxidative stress and inflammation, the initiation of structural and functional remodelling in the cardiovascular system, the promotion of exerkine secretion from skeletal muscles and other tissues, and decreases in the risk factors for cardiovascular disease.

**Figure 3:** Long-term moderate- and high-intensity exercise induces cardiovascular remodelling: Moderate- and high-intensity exercise performed over a prolonged period both causes and promotes structural and functional remodelling in the cardiovascular system. The structural remodeling process involves physiological cardiac hypertrophy, a decrease in the vascular wall thickness, and increases in the luminal width of conduit arteries. The process of functional remodelling is characterized by increases in cardiac contraction and dilatation and reductions in the heart rate and blood pressure.

**Figure 4:** Exercise induces multiple tissues to produce and release exerkines, which mediate cardiovascular protection: Through the mediation of cell-to-cell contacts and crosstalk between organs and tissues, exercise enhances cardiovascular health by inducing the production of exerkines in several different tissues. Among the primary carriers of miRNAs and other exerkines are exosomes.

## Data Availability

Not applicable.

## Abbreviations

Proliferator-activated receptor-coactivator-1 (PCC-1), metabolic problem of basal and branched-amino acids (BCAAs), reactive oxygen species (ROS), non-communicable diseases (NCDs), C-reactive protein (hS-CRP), interleukin-6 (IL-6), necrosis factor-α (TNF-α), interleukin-1 (IL-1), Insulin-like growth factor 1 (IGF1), Nitric oxide (NO), High-density lipoprotein cholesterol (HDL-c), Heart rate variability (HRV), Cardiorespiratory fitness (CRF), Metabolic equivalent (MET), fibronectin type III domain-containing protein 5 (FNDC5), Uncoupling protein-1 (UCP-1), Meteorin-like protein (METRNL), Follistatin like 1 (FSTL1), Long noncoding RNA (lncRNA), Heart failure (HF).

The article "Cardiovascular Disease and Exercise: From Molecular Mechanisms to Clinical Applications" was retracted in 2023. Reason: plagiarism.

## References

[1] Lavie C.J., Ozemek C., Carbone S., Katzmarzyk P.T., Blair S.N. (2019). Sedentary Behavior, Exercise, and Cardiovascular Health. Circ. Res..

[2] Kramer A. (2020). An Overview of the Beneficial Effects of Exercise on Health and Performance. Adv. Exp. Med. Biol..

[3] Coats A.J.S., Forman D.E., Haykowsky M., Kitzman D.W., McNeil A., Campbell T.S., Arena R. (2017). Physical function and exercise training in older patients with heart failure. Nat. Rev. Cardiol..

[4] Zhang G.L., Sun M.L., Zhang X.A. (2021). Exercise-Induced Adult Cardiomyocyte Proliferation in Mammals. Front. Physiol..

[5] Wang Y., Tian Z., Zang W., Jiang H., Li Y., Wang S., Chen S. (2015). Exercise training reduces insulin resistance in postmyocardial infarction rats. Physiol. Rep..

[6] Jia D., Hou L., Lv Y., Xi L., Tian Z. (2019). Postinfarction exercise training alleviates cardiac dysfunction and adverse remodeling via mitochondrial biogenesis and SIRT1/PGC-1alpha/PI3K/Akt signaling. J. Cell. Physiol..

[7] Neri Serneri G.G., Boddi M., Modesti P.A., Cecioni I., Coppo M., Padeletti L., Michelucci A., Colella A., Galanti G. (2001). Increased cardiac sympathetic activity and insulin-like growth factor-I formation are associated with physiological hypertrophy in athletes. Circ. Res..

[8] Lavie C.J., Arena R., Swift D.L., Johannsen N.M., Sui X., Lee D.C., Earnest C.P., Church T.S., O’Keefe J.H., Milani R.V. (2015). Exercise and the cardiovascular system: Clinical science and cardiovascular outcomes. Circ. Res..

[9] Guo Y., Wang S., Liu Y., Fan L., Booz G.W., Roman R.J., Chen Z., Fan F. (2020). Accelerated cerebral vascular injury in diabetes is associated with vascular smooth muscle cell dysfunction. Geroscience.

[10] Short K.R., Chadwick J.Q., Teague A.M., Tullier M.A., Wolbert L., Coleman C., Copeland K.C. (2019). Effect of Obesity and Exercise Training on Plasma Amino Acids and Amino Metabolites in American Indian Adolescents. J. Clin. Endocrinol. Metab..

[11] Umpierre D., Ribeiro P.A., Kramer C.K., Leitao C.B., Zucatti A.T., Azevedo M.J., Gross J.L., Ribeiro J.P., Schaan B.D. (2011). Physical activity advice only or structured exercise training and association with HbA1c levels in type 2 diabetes: A systematic review and meta-analysis. JAMA.

The article "Cardiovascular Disease and Exercise: From Molecular Mechanisms to Clinical Applications" was retracted in 2023. Reason: plagiarism.

[12] Li Y., Xiong Z., Yan W., Gao E., Cheng H., Wu G., Liu Y., Zhang L., Li C., Wang S. (2020). Branched chain amino acids exacerbate myocardial ischemia/reperfusion vulnerability via enhancing GCN2/ATF6/PPAR-alpha pathway-dependent fatty acid oxidation. Theranostics.

[13] Murthy V.L., Yu B., Wang W., Zhang X., Alkis T., Pico A.R., Yeri A., Bhupathiraju S.N., Bressler J., Ballantyne C.M. (2020). Molecular Signature of Multisystem Cardiometabolic Stress and Its Association with Prognosis. JAMA Cardiol..

[14] Shaw E., Leung G.K.W., Jong J., Coates A.M., Davis R., Blair M., Huggins C.E., Dorrian J., Banks S., Kellow N.J. (2019). The Impact of Time of Day on Energy Expenditure: Implications for Long-Term Energy Balance. Nutrients.

[15] Powers S.K., Deminice R., Ozdemir M., Yoshihara T., Bomkamp M.P., Hyatt H. (2020). Exercise-induced oxidative stress: Friend or foe?. J. Sport Health Sci..

[16] Jackson M.J. (2011). Control of reactive oxygen species production in contracting skeletal muscle. Antioxid. Redox Signal..

[17] Taherkhani S., Suzuki K., Castell L. (2020). A Short Overview of Changes in Inflammatory Cytokines and Oxidative Stress in Response to Physical Activity and Antioxidant Supplementation. Antioxidants.

[18] Ristow M., Zarse K., Oberbach A., Kloting N., Birringer M., Kiehntopf M., Stumvoll M., Kahn C.R., Bluher M. (2009). Antioxidants prevent health-promoting effects of physical exercise in humans. Proc. Natl. Acad. Sci. USA.

[19] Ghahremani R., Damirchi A., Salehi I., Komaki A., Esposito F. (2018). Mitochondrial dynamics as an underlying mechanism involved in aerobic exercise training-induced cardioprotection against ischemia-reperfusion injury. Life Sci..

[20] Powers S.K., Sollanek K.J., Wiggs M.P., Demirel H.A., Smuder A.J. (2014). Exercise-induced improvements in myocardial antioxidant capacity: The antioxidant players and cardioprotection. Free Radic. Res..

[21] Done A.J., Traustadottir T. (2016). Nrf2 mediates redox adaptations to exercise. Redox Biol..

[22] Milani R.V., Lavie C.J., Mehra M.R. (2004). Reduction in C-reactive protein through cardiac rehabilitation and exercise training. J. Am. Coll. Cardiol..

[23] Starkie R., Ostrowski S.R., Jauffred S., Febbraio M., Pedersen B.K. (2003). Exercise and IL-6 infusion inhibit endotoxin-induced TNF-alpha production in humans. FASEB J..

[24] Mathur N., Pedersen B.K. (2008). Exercise as a mean to control low-grade systemic inflammation. Mediat. Inflamm..

[25] Rysz J., Franczyk B., Rysz-Gorzynska M., Gluba-Brzozka A. (2021). Ageing, Age-Related Cardiovascular Risk and the Beneficial Role of Natural Components Intake. Int. J. Mol. Sci..

The article "Cardiovascular Disease and Exercise: From Molecular Mechanisms to Clinical Applications" was retracted in 2023. Reason: plagiarism.

[26] Szalewska D., Radkowski M., Demkow U., Winklewski P.J. (2017). Exercise Strategies to Counteract Brain Aging Effects. Adv. Exp. Med. Biol..

[27] Janssen J.A. (2016). Impact of Physical Exercise on Endocrine Aging. Front. Horm. Res..

[28] Leosco D., Parisi V., Femminella G.D., Formisano R., Petraglia L., Allocca E., Bonaduce D. (2013). Effects of exercise training on cardiovascular adrenergic system. Front. Physiol..

[29] Baekkerud F.H., Salerno S., Ceriotti P., Morland C., Storm-Mathisen J., Bergersen L.H., Hoydal M.A., Catalucci D., Stolen T.O. (2019). High Intensity Interval Training Ameliorates Mitochondrial Dysfunction in the Left Ventricle of Mice with Type 2 Diabetes. Cardiovasc. Toxicol..

[30] Roh J., Rhee J., Chaudhari V., Rosenzweig A. (2016). The Role of Exercise in Cardiac Aging: From Physiology to Molecular Mechanisms. Circ. Res..

[31] Gliemann L., Nyberg M., Hellsten Y. (2016). Effects of exercise training and resveratrol on vascular health in aging. Free Radic. Biol. Med..

[32] Radak Z., Torma F., Berkes I., Goto S., Mimura T., Posa A., Balogh L., Boldogh I., Suzuki K., Higuchi M. (2019). Exercise effects on physiological function during aging. Free Radic. Biol. Med..

[33] Naci H., Salcher-Konrad M., Dias S., Blum M.R., Sahoo S.A., Nunan D., Ioannidis J.P.A. (2019). How does exercise treatment compare with antihypertensive medications? A network meta-analysis of 391 randomised controlled trials assessing exercise and medication effects on systolic blood pressure. Br. J. Sports Med..

[34] Costa E.C., Hay J.L., Kehler D.S., Boreskie K.F., Arora R.C., Umpierre D., Szwajcer A., Duhamel T.A. (2018). Effects of High-Intensity Interval Training Versus Moderate-Intensity Continuous Training on Blood Pressure in Adults with Pre- to Established Hypertension: A Systematic Review and Meta-Analysis of Randomized Trials. Sports Med..

[35] Ciolac E.G., Bocchi E.A., Bortolotto L.A., Carvalho V.O., Greve J.M., Guimaraes G.V. (2010). Effects of high-intensity aerobic interval training vs. moderate exercise on hemodynamic, metabolic and neuro-humoral abnormalities of young normotensive women at high familial risk for hypertension. Hypertens. Res..

[36] Feraco A., Gorini S., Armani A., Camajani E., Rizzo M., Caprio M. (2021). Exploring the Role of Skeletal Muscle in Insulin Resistance: Lessons from Cultured Cells to Animal Models. Int. J. Mol. Sci..

[37] Powers S.K., Morton A.B., Ahn B., Smuder A.J. (2016). Redox control of skeletal muscle atrophy. Free Radic. Biol. Med..

[38] Kokkinidis D.G., Arfaras-Melainis A., Giannakoulas G. (2021). Sarcopenia in heart failure: ‘waste’ the appropriate time and resources, not the muscles. Eur. J. Prev. Cardiol..

The article "Cardiovascular Disease and Exercise: From Molecular Mechanisms to Clinical Applications" was retracted in 2023. Reason: plagiarism.

[39] Konishi M., Kagiyama N., Kamiya K., Saito H., Saito K., Ogasahara Y., Maekawa E., Misumi T., Kitai T., Iwata K. (2021). Impact of sarcopenia on prognosis in patients with heart failure with reduced and preserved ejection fraction. Eur. J. Prev. Cardiol..

[40] Son J., Jang L.G., Kim B.Y., Lee S., Park H. (2020). The Effect of Athletes’ Probiotic Intake May Depend on Protein and Dietary Fiber Intake. Nutrients.

[41] Allen J.M., Mailing L.J., Niemiro G.M., Moore R., Cook M.D., White B.A., Holscher H.D., Woods J.A. (2018). Exercise Alters Gut Microbiota Composition and Function in Lean and Obese Humans. Med. Sci. Sports Exerc..

[42] Barton W., Penney N.C., Cronin O., Garcia-Perez I., Molloy M.G., Holmes E., Shanahan F., Cotter P.D., O’Sullivan O. (2018). The microbiome of professional athletes differs from that of more sedentary subjects in composition and particularly at the functional metabolic level. Gut.

[43] Liu Y., Wang Y., Ni Y., Cheung C.K.Y., Lam K.S.L., Wang Y., Xia Z., Ye D., Guo J., Tse M.A. (2020). Gut Microbiome Fermentation Determines the Efficacy of Exercise for Diabetes Prevention. Cell Metab..

[44] Lavie C.J., Milani R.V. (2004). Prevalence of anxiety in coronary patients with improvement following cardiac rehabilitation and exercise training. Am. J. Cardiol..

[45] Hambrecht R., Walther C., Mobius-Winkler S., Gielen S., Linke A., Conradi K., Erbs S., Kluge R., Kendziorra K., Sabri O. (2004). Percutaneous coronary angioplasty compared with exercise training in patients with stable coronary artery disease: A randomized trial. Circulation.

[46] Thijssen D.H., Cable N.T., Green D.J. (2012). Impact of exercise training on arterial wall thickness in humans. Clin. Sci..

[47] Shimada K., Mikami Y., Murayama T., Yokode M., Fujita M., Kita T., Kishimoto C. (2011). Atherosclerotic plaques induced by marble-burying behavior are stabilized by exercise training in experimental atherosclerosis. Int. J. Cardiol..

[48] Seals D.R., Desouza C.A., Donato A.J., Tanaka H. (2008). Habitual exercise and arterial aging. J. Appl. Physiol..

[49] Schuttler D., Clauss S., Weckbach L.T., Brunner S. (2019). Molecular Mechanisms of Cardiac Remodeling and Regeneration in Physical Exercise. Cells.

[50] Golbidi S., Laher I. (2011). Molecular mechanisms in exercise-induced cardioprotection. Cardiol. Res. Pract..

[51] Gu J.W., Gadonski G., Wang J., Makey I., Adair T.H. (2004). Exercise increases endostatin in circulation of healthy volunteers. BMC Physiol..

[52] Heaps C.L., Robles J.C., Sarin V., Mattox M.L., Parker J.L. (2014). Exercise training-induced adaptations in mediators of sustained endothelium-dependent coronary artery relaxation in a porcine model of ischemic heart disease. Microcirculation.

The article "Cardiovascular Disease and Exercise: From Molecular Mechanisms to Clinical Applications" was retracted in 2023. Reason: plagiarism.

[53] Green D.J., O’Driscoll G., Joyner M.J., Cable N.T. (2008). Exercise and cardiovascular risk reduction: Time to update the rationale for exercise?. J. Appl. Physiol..

[54] Hambrecht R., Adams V., Erbs S., Linke A., Krankel N., Shu Y., Baither Y., Gielen S., Thiele H., Gummert J.F. (2003). Regular physical activity improves endothelial function in patients with coronary artery disease by increasing phosphorylation of endothelial nitric oxide synthase. Circulation.

[55] Hou Z., Qin X., Hu Y., Zhang X., Li G., Wu J., Li J., Sha J., Chen J., Xia J. (2019). Longterm Exercise-Derived Exosomal miR-342-5p: A Novel Exerkine for Cardioprotection. Circ. Res..

[56] Ko J., Deprez D., Shaw K., Alcorn J., Hadjistavropoulos T., Tomczak C., Foulds H., Chilibeck P.D. (2021). Stretching is Superior to Brisk Walking for Reducing Blood Pressure in People with High-Normal Blood Pressure or Stage I Hypertension. J. Phys. Act. Health.

[57] Beech D.J., Kalli A.C. (2019). Force Sensing by Piezo Channels in Cardiovascular Health and Disease. Arterioscler. Thromb. Vasc. Biol..

[58] Shah V., Patel S., Shah J. (2022). Emerging role of Piezo ion channels in cardiovascular development. Dev. Dyn..

[59] Golbidi S., Laher I. (2012). Exercise and the cardiovascular system. Cardiol. Res. Pract..

[60] Young C.G., Knight C.A., Vickers K.C., Westbrook D., Madamanchi N.R., Runge M.S., Ischiropoulos H., Ballinger S.W. (2005). Differential effects of exercise on aortic mitochondria. Am. J. Physiol. Heart Circ. Physiol..

[61] Fulghum K., Hill B.G. (2018). Metabolic Mechanisms of Exercise-Induced Cardiac Remodeling. Front. Cardiovasc. Med..

[62] Gibb A.A., Epstein P.N., Uchida S., Zheng Y., McNally L.A., Obal D., Katragadda K., Trainor P., Conklin D.J., Brittian K.R. (2017). Exercise-Induced Changes in Glucose Metabolism Promote Physiological Cardiac Growth. Circulation.

[63] Lee Y., Min K., Talbert E.E., Kavazis A.N., Smuder A.J., Willis W.T., Powers S.K. (2012). Exercise protects cardiac mitochondria against ischemia-reperfusion injury. Med. Sci. Sports Exerc..

[64] Boulghobra D., Coste F., Geny B., Reboul C. (2020). Exercise training protects the heart against ischemia-reperfusion injury: A central role for mitochondria?. Free Radic. Biol. Med..

[65] Seals D.R., Dinenno F.A. (2004). Collateral damage: Cardiovascular consequences of chronic sympathetic activation with human aging. Am. J. Physiol. Heart Circ. Physiol..

[66] DeFina L.F., Haskell W.L., Willis B.L., Barlow C.E., Finley C.E., Levine B.D., Cooper K.H. (2015). Physical activity versus cardiorespiratory fitness: Two (partly) distinct components of cardiovascular health?. Prog. Cardiovasc. Dis..

The article "Cardiovascular Disease and Exercise: From Molecular Mechanisms to Clinical Applications" was retracted in 2023. Reason: plagiarism.

[67] Myers J., McAuley P., Lavie C.J., Despres J.P., Arena R., Kokkinos P. (2015). Physical activity and cardiorespiratory fitness as major markers of cardiovascular risk: Their independent and interwoven importance to health status. Prog. Cardiovasc. Dis..

[68] Safdar A., Saleem A., Tarnopolsky M.A. (2016). The potential of endurance exercise-derived exosomes to treat metabolic diseases. Nat. Rev. Endocrinol..

[69] Heineke J., Auger-Messier M., Xu J., Sargent M., York A., Welle S., Molkentin J.D. (2010). Genetic deletion of myostatin from the heart prevents skeletal muscle atrophy in heart failure. Circulation.

[70] Biesemann N., Mendler L., Wietelmann A., Hermann S., Schafers M., Kruger M., Boettger T., Borchardt T., Braun T. (2014). Myostatin regulates energy homeostasis in the heart and prevents heart failure. Circ. Res..

[71] Nara H., Watanabe R. (2021). Anti-Inflammatory Effect of Muscle-Derived Interleukin-6 and Its Involvement in Lipid Metabolism. Int. J. Mol. Sci..

[72] Ricard N., Tu L., Le Hiress M., Huertas A., Phan C., Thuillet R., Sattler C., Fadel E., Seferian A., Montani D. (2014). Increased pericyte coverage mediated by endothelial-derived fibroblast growth factor-2 and interleukin-6 is a source of smooth muscle-like cells in pulmonary hypertension. Circulation.

[73] Kolak A., Kaminska M., Wysokinska E., Surdyka D., Kieszko D., Pakiela M., Burdan F. (2017). The problem of fatigue in patients suffering from neoplastic disease. Contemp. Oncol..

[74] Zhou X., Xu M., Bryant J.L., Ma J., Xu X. (2019). Exercise-induced myokine FNDC5/irisin functions in cardiovascular protection and intracerebral retrieval of synaptic plasticity. Cell Biosci..

[75] Rao R.R., Long J.Z., White J.P., Svensson K.J., Lou J., Lokurkar I., Jedrychowski M.P., Ruas J.L., Wrann C.D., Lo J.C. (2014). Meteorin-like is a hormone that regulates immune-adipose interactions to increase beige fat thermogenesis. Cell.

[76] Zhong J.C., Zhang Z.Z., Wang W., McKinnie S.M.K., Vederas J.C., Oudit G.Y. (2017). Targeting the apelin pathway as a novel therapeutic approach for cardiovascular diseases. Biochim. Biophys. Acta Mol. Basis Dis..

[77] Ouchi N., Oshima Y., Ohashi K., Higuchi A., Ikegami C., Izumiya Y., Walsh K. (2008). Follistatin-like 1, a secreted muscle protein, promotes endothelial cell function and revascularization in ischemic tissue through a nitric-oxide synthase-dependent mechanism. J. Biol. Chem..

[78] Reynolds J.C., Lai R.W., Woodhead J.S.T., Joly J.H., Mitchell C.J., Cameron-Smith D., Lu R., Cohen P., Graham N.A., Benayoun B.A. (2021). MOTS-c is an exercise-induced mitochondrial-encoded regulator of age-dependent physical decline and muscle homeostasis. Nat. Commun..

The article "Cardiovascular Disease and Exercise: From Molecular Mechanisms to Clinical Applications" was retracted in 2023. Reason: plagiarism.

[79] Roberts L.D., Bostrom P., O’Sullivan J.F., Schinzel R.T., Lewis G.D., Dejam A., Lee Y.K., Palma M.J., Calhoun S., Georgiadi A. (2014). beta-Aminoisobutyric acid induces browning of white fat and hepatic beta-oxidation and is inversely correlated with cardiometabolic risk factors. Cell Metab..

[80] Moschen A.R., Wieser V., Tilg H. (2012). Adiponectin: Key player in the adipose tissue-liver crosstalk. Curr. Med. Chem..

[81] Ouchi N., Shibata R., Walsh K. (2006). Cardioprotection by adiponectin. Trends Cardiovasc. Med..

[82] Aljafary M.A., Al-Suhaimi E.A. (2022). Adiponectin System (Rescue Hormone): The Missing Link between Metabolic and Cardiovascular Diseases. Pharmaceutics.

[83] Mattu H.S., Randeva H.S. (2013). Role of adipokines in cardiovascular disease. J. Endocrinol..

[84] Ma S., Liao Y. (2019). Noncoding RNAs in exercise-induced cardio-protection for chronic heart failure. EBioMedicine.

[85] Wu G., Zhang X., Gao F. (2021). The epigenetic landscape of exercise in cardiac health and disease. J. Sport Health Sci..

[86] Nielsen S., Scheele C., Yfanti C., Akerstrom T., Nielsen A.R., Pedersen B.K., Laye M.J. (2010). Muscle specific microRNAs are regulated by endurance exercise in human skeletal muscle. J. Physiol..

[87] Radom-Aizik S., Zaldivar F., Oliver S., Galassetti P., Cooper D.M. (2010). Evidence for microRNA involvement in exercise-associated neutrophil gene expression changes. J. Appl. Physiol..

[88] Ma Z., Qi J., Meng S., Wen B., Zhang J. (2013). Swimming exercise training-induced left ventricular hypertrophy involves microRNAs and synergistic regulation of the PI3K/AKT/mTOR signaling pathway. Eur. J. Appl. Physiol..

[89] DA Silva N.D., Fernandes T., Soci U.P., Monteiro A.W., Phillips M.I., de Oliveira E.M. (2012). Swimming training in rats increases cardiac MicroRNA-126 expression and angiogenesis. Med. Sci. Sports Exerc..

[90] Melo S.F., Barauna V.G., Neves V.J., Fernandes T., Lara Lda S., Mazzotti D.R., Oliveira E.M. (2015). Exercise training restores the cardiac microRNA-1 and -214 levels regulating Ca2+ handling after myocardial infarction. BMC Cardiovasc. Disord..

[91] Melo S.F., Fernandes T., Barauna V.G., Matos K.C., Santos A.A., Tucci P.J., Oliveira E.M. (2014). Expression of MicroRNA-29 and Collagen in Cardiac Muscle after Swimming Training in Myocardial-Infarcted Rats. Cell Physiol. Biochem..

[92] Liu S.X., Zheng F., Xie K.L., Xie M.R., Jiang L.J., Cai Y. (2019). Exercise Reduces Insulin Resistance in Type 2 Diabetes Mellitus via Mediating the lncRNA MALAT1/MicroRNA-382-3p/Resistin Axis. Mol. Ther. Nucleic Acids.

[93] Jia G., DeMarco V.G., Sowers J.R. (2016). Insulin resistance and hyperinsulinaemia in diabetic cardiomyopathy. Nat. Rev. Endocrinol..

The article "Cardiovascular Disease and Exercise: From Molecular Mechanisms to Clinical Applications" was retracted in 2023. Reason: plagiarism.

[94] Adeva-Andany M.M., Martinez-Rodriguez J., Gonzalez-Lucan M., Fernandez-Fernandez C., Castro-Quintela E. (2019). Insulin resistance is a cardiovascular risk factor in humans. Diabetol. Metab. Syndr..

[95] Iaccarino G., Franco D., Sorriento D., Strisciuglio T., Barbato E., Morisco C. (2021). Modulation of Insulin Sensitivity by Exercise Training: Implications for Cardiovascular Prevention. J. Cardiovasc. Transl. Res..

[96] Nasi M., Patrizi G., Pizzi C., Landolfo M., Boriani G., Dei Cas A., Cicero A.F.G., Fogacci F., Rapezzi C., Sisca G. (2019). The role of physical activity in individuals with cardiovascular risk factors: An opinion paper from Italian Society of Cardiology-Emilia Romagna-Marche and SIC-Sport. J. Cardiovasc. Med..

[97] Hawley J.A., Lessard S.J. (2008). Exercise training-induced improvements in insulin action. Acta Physiol..

[98] Borghouts L.B., Keizer H.A. (2000). Exercise and insulin sensitivity: A review. Int. J. Sports Med..

[99] Grunewald Z.I., Ramirez-Perez F.I., Woodford M.L., Morales-Quinones M., Mejia S., Manrique-Acevedo C., Siebenlist U., Martinez-Lemus L.A., Chandrasekar B., Padilla J. (2020). TRAF3IP2 (TRAF3 Interacting Protein 2) Mediates Obesity-Associated Vascular Insulin Resistance and Dysfunction in Male Mice. Hypertension.

[100] Saotome M., Ikoma T., Hasan P., Maekawa Y. (2019). Cardiac Insulin Resistance in Heart Failure: The Role of Mitochondrial Dynamics. Int. J. Mol. Sci..

[101] Fu F., Zhao K., Li J., Xu J., Zhang Y., Liu C., Yang W., Gao C., Li J., Zhang H. (2015). Direct Evidence that Myocardial Insulin Resistance following Myocardial Ischemia Contributes to Post-Ischemic Heart Failure. Sci. Rep..

[102] Xing W., Yan W., Liu P., Ji L., Li Y., Sun L., Tao L., Zhang H., Gao F. (2013). A novel mechanism for vascular insulin resistance in normotensive young SHRs: Hypoadiponectinemia and resultant APPL1 downregulation. Hypertension.

[103] Zhang K.R., Liu H.T., Zhang H.F., Zhang Q.J., Li Q.X., Yu Q.J., Guo W.Y., Wang H.C., Gao F. (2007). Long-term aerobic exercise protects the heart against ischemia/reperfusion injury via PI3 kinase-dependent and Akt-mediated mechanism. Apoptosis.

[104] Zhang Q.J., Li Q.X., Zhang H.F., Zhang K.R., Guo W.Y., Wang H.C., Zhou Z., Cheng H.P., Ren J., Gao F. (2007). Swim training sensitizes myocardial response to insulin: Role of Akt-dependent eNOS activation. Cardiovasc. Res..

[105] Frasier C.R., Moore R.L., Brown D.A. (2011). Exercise-induced cardiac preconditioning: How exercise protects your achy-breaky heart. J. Appl. Physiol..

[106] Del Buono M.G., Arena R., Borlaug B.A., Carbone S., Canada J.M., Kirkman D.L., Garten R., Rodriguez-Miguelez P., Guazzi M., Lavie C.J. (2019). Exercise Intolerance in Patients with Heart Failure: JACC State-of-the-Art Review. J. Am. Coll. Cardiol..

The article "Cardiovascular Disease and Exercise: From Molecular Mechanisms to Clinical Applications" was retracted in 2023. Reason: plagiarism.

[107] Houstis N.E., Eisman A.S., Pappagianopoulos P.P., Wooster L., Bailey C.S., Wagner P.D., Lewis G.D. (2018). Exercise Intolerance in Heart Failure with Preserved Ejection Fraction: Diagnosing and Ranking Its Causes Using Personalized O_2_ Pathway Analysis. Circulation.

[108] Dhakal B.P., Malhotra R., Murphy R.M., Pappagianopoulos P.P., Baggish A.L., Weiner R.B., Houstis N.E., Eisman A.S., Hough S.S., Lewis G.D. (2015). Mechanisms of exercise intolerance in heart failure with preserved ejection fraction: The role of abnormal peripheral oxygen extraction. Circ. Heart Fail..

[109] Pelliccia A., Sharma S., Gati S., Back M., Borjesson M., Caselli S., Collet J.P., Corrado D., Drezner J.A., Halle M. (2021). 2020 ESC Guidelines on sports cardiology and exercise in patients with cardiovascular disease. Eur. Heart J..

[110] Guazzi M., Arena R., Halle M., Piepoli M.F., Myers J., Lavie C.J. (2016). 2016 Focused Update: Clinical Recommendations for Cardiopulmonary Exercise Testing Data Assessment in Specific Patient Populations. Circulation.

[111] Ismail H., McFarlane J.R., Nojoumian A.H., Dieberg G., Smart N.A. (2013). Clinical outcomes and cardiovascular responses to different exercise training intensities in patients with heart failure: A systematic review and meta-analysis. JACC Heart Fail..

[112] Gomes Neto M., Duraes A.R., Conceicao L.S.R., Saquetto M.B., Ellingsen O., Carvalho V.O. (2018). High intensity interval training versus moderate intensity continuous training on exercise capacity and quality of life in patients with heart failure with reduced ejection fraction: A systematic review and meta-analysis. Int. J. Cardiol..

[113] Piccini J.P., Hellkamp A.S., Whellan D.J., Ellis S.J., Keteyian S.J., Kraus W.E., Hernandez A.F., Daubert J.P., Pina L., O’Connor C.M. (2013). Exercise training and implantable cardioverter-defibrillator shocks in patients with heart failure: Results from HF-ACTION (Heart Failure and A Controlled Trial Investigating Outcomes of Exercise TraiNing). JACC Heart Fail..

[114] Schindler M.J., Adams V., Halle M. (2019). Exercise in Heart Failure-What Is the Optimal Dose to Improve Pathophysiology and Exercise Capacity?. Curr. Heart Fail. Rep..

[115] Harwood A.E., Russell S., Okwose N.C., McGuire S., Jakovljevic D.G., McGregor G. (2021). A systematic review of rehabilitation in chronic heart failure: Evaluating the reporting of exercise interventions. ESC Heart Fail..

[116] Fukuta H., Goto T., Wakami K., Kamiya T., Ohte N. (2021). Effect of renin-angiotensin system inhibition on cardiac structure and function and exercise capacity in heart failure with preserved ejection fraction: A meta-analysis of randomized controlled trials. Heart Fail. Rev..

The article "Cardiovascular Disease and Exercise: From Molecular Mechanisms to Clinical Applications" was retracted in 2023. Reason: plagiarism.

[117] Marinus N., Hansen D., Feys P., Meesen R., Timmermans A., Spildooren J. (2019). The Impact of Different Types of Exercise Training on Peripheral Blood Brain-Derived Neurotrophic Factor Concentrations in Older Adults: A Meta-Analysis. Sports Med..

[118] Vona M., Codeluppi G.M., Iannino T., Ferrari E., Bogousslavsky J., von Segesser L.K. (2009). Effects of different types of exercise training followed by detraining on endothelium-dependent dilation in patients with recent myocardial infarction. Circulation.

[119] Oja P., Kelly P., Pedisic Z., Titze S., Bauman A., Foster C., Hamer M., Hillsdon M., Stamatakis E. (2017). Associations of specific types of sports and exercise with all-cause and cardiovascular-disease mortality: A cohort study of 80 306 British adults. Br. J. Sports Med..

[120] Strain T., Wijndaele K., Dempsey P.C., Sharp S.J., Pearce M., Jeon J., Lindsay T., Wareham N., Brage S. (2020). Wearable-device-measured physical activity and future health risk. Nat. Med..

[121] Savikj M., Gabriel B.M., Alm P.S., Smith J., Caidahl K., Bjornholm M., Fritz T., Krook A., Zierath J.R., Wallberg-Henriksson H. (2019). Afternoon exercise is more efficacious than morning exercise at improving blood glucose levels in individuals with type 2 diabetes: A randomised crossover trial. Diabetologia.

[122] Fernandes R.A., Zanesco A. (2010). Early physical activity promotes lower prevalence of chronic diseases in adulthood. Hypertens. Res..

[123] Harris J.E., Baer L.A., Stanford K.I. (2018). Maternal Exercise Improves the Metabolic Health of Adult Offspring. Trends Endocrinol. Metab..

[124] Stanford K.I., Takahashi H., So K., Alves-Wagner A.B., Prince N.B., Lehnig A.C., Getchell K.M., Lee M.Y., Hirshman M.F., Goodyear L.J. (2017). Maternal Exercise Improves Glucose Tolerance in Female Offspring. Diabetes.

[125] Stanford K.I., Rasmussen M., Baer L.A., Lehnig A.C., Rowland L.A., White J.D., So K., De Sousa-Coelho A.L., Hirshman M.F., Patti M.E. (2018). Paternal Exercise Improves Glucose Metabolism in Adult Offspring. Diabetes.

